RETRACTED

# Therapeutic Effect Analysis of Plasma Bipolar Intelligent Electrotonic for Cystostomy in the Treatment of Senile Prostatic Hyperplasia

**DOI:** 10.1155/2021/9332848

**Published:** 2021-10-15

**Authors:** Zhixin You, Haoyu Zhang, Xiaoxiang Zhang, Yilei Li

**Affiliations:** The Second People's Hospital of Kunshan, Jiangsu Kunshan 215300, China

## Abstract

To solve prostatic hyperplasia in the elderly, a method of cystostomy with plasma bipolar resection was proposed. From January 2019 to March 2020, 42 patients with BPH who needed surgical treatment in the urological department were selected. Cystostomy was performed in bipolar TURP. The cystostomy group and robot group were divided into two groups. The surgical safety, surgical efficiency, complications, and nursing time between the two groups were compared. The results showed that the experimental and control groups' RUV values were significantly lower than those before surgery. In comparison, the Qmax value was considerably higher than that before surgery. The difference was statistically significant (*P* < 0.05), suggesting that the cystostomy group in bipolar TURP had more substantial improvement of dysuria, better recovery of detrusor function, and better prognosis. It was proved that, for BPH below 80 g, cystostomy could reduce the operation time, bladder irrigation time, catheter indwelling time, and postoperative hospital stay, improve the operation efficiency, and have the same effect on patients' symptoms improvement, more excellent psychological support, and higher quality of life score. It is proved that plasma bipolar resection combined with cystostomy can effectively improve annual BPH surgery.

## 1. Introduction

Benign prostatic hyperplasia (BPH) is a common disease in older men. By the age of 60, more than half of men have BPH. By the age of 80, almost all men have BPH [1]. It often leads to lower urinary tract symptoms such as dysuria, frequent urination, urgent urination, and increased nocturia, which seriously affects the life health and quality of life of older men. Traditional unipolar transurethral resection of the prostate (unipolar TURP) is the “gold standard” for surgical treatment of benign prostatic hyperplasia [2]. However, because the lavage fluid used in unipolar TURP is nonconductive nonionic fluid, excessive absorption of this nonionic fluid during the operation may cause transurethral resection syndrome (TURS), mainly characterized by diluent hyponatremia and hypervolume, which seriously threatens the life safety of patients [3]. Simultaneous intraoperative cystostomy can reduce the absorption of lavage fluid during unipolar TURP and thus prevent the occurrence of TURS [4]. As one of the methods of “low-pressure lavage technique,” many domestic kinds of literature have reported that unipolar TURP combined with cystostomy has a lot of benefits, such as shortening operation time, reducing intraoperative blood loss, reducing the incidence of TURS, and increasing the safety of high-risk patients [5]. However, for bipolar TURP, especially for bipolar TURP < 80 GBPH, the benefits and necessity of cystostomy have been rarely discussed and reported. Compared with unipolar TURP, bipolar transurethral resection of the prostate (bipolar TURP) has a lower incidence of TURS and other complications [6], shaking the status of traditional unipolar TURP. Therefore, it is necessary to discuss whether concurrent cystostomy is still of obvious benefit and necessity under the premise of bipolar TURP, especially for bipolar TURP with BPH below 80 g. By retrospectively analyzing the case data of patients with BPH below 80 g treated with bipolar TURP in our hospital since January 2018, the benefits and necessity of cystostomy were discussed to provide clinical reference for clinical workers cystostomy should be combined with bipolar TURP treatment in our hospital.

RETRACTED

Therefore, studies at home and abroad continue. Ma et al. investigate the application effect of transurethral plasma resection or bipolar plasma resection in treating senile prostatic hyperplasia (BPH) [7]. Crucittiet al. discussed the surgical methods and efficacy of transurethral bipolar plasma resection (PKRP) in treating prostatic hyperplasia [8]. Bhojaniet al. retrospectively analyzed the clinical data of 83 elderly patients with high-risk bulk-size prostatic hyperplasia treated by transurethral plasma resection for 1 to 12 months of follow-up. The international prostate symptom score (IPSS), quality of life (QOL), maximum urine flow rate (Qmax), and residual urine volume (RUV) were significantly improved compared with those before operation, and all patients completed the operation safely without complications such as transurethral resection syndrome and urinary incontinence [9]. We treated bladder stones first and then performed plasma resection of the prostate through the urethra, without urethral or bladder bleeding. In this way, the operation can be carried out smoothly, the operation time can be shortened, and electrosurgical syndrome can be avoided [10]. Based on existing research, this article proposes a new method of plasma-directed bipolar resection for cystostomy. Forty-two patients with BPH who were admitted to the department of urology of a hospital from January 2018 to March 2019 and required surgical treatment were selected. According to whether cystostomy was performed during bipolar TURP, the patients were divided into the cystostomy group and robot group, and the surgical safety, surgical efficiency, complications, and nursing time were compared between the two groups. The results showed that the RUV value of the experimental group and the control group was significantly lower than that before surgery, while the Qmax value was considerably higher than that before surgery, and the difference was statistically significant (*P* < 0.05), suggesting that the cystostomy group in bipolar TURP had more substantial improvement of dysuria, better recovery of detrusor function, and better prognosis. It was proved that, for BPH below 80 g, cystostomy could reduce the operation time, bladder irrigation time, catheter indwelling time, and postoperative hospital stay, improve the operation efficiency, and have the same effect on patients' symptoms improvement, excellent psychological support, and higher quality of life score. It is proved that plasma bipolar electroreception combined with cystostomy can effectively solve and improve the surgical effect of annual prostatic hyperplasia.

RETRACTED

## 2. Materials and Methods

### 2.1. Selection of Objects

From January 2019 to March 2020, 42 patients with BPH who needed surgical treatment in the urological department were selected. The age was 61∼79 years (mean 73 years old), and the prostate volume measured by B-ultrasound was 43.3∼79.8 mL (prostate volume: prostate length × width × height × 0.52). There were 26 patients in the experimental group, aged 61∼79 years, with an average of 71 years. The prostate volume was 43.3∼73.8 mL, with an average of 53.6 mL. In the control group, 16 patients (age 61∼77 years old, average 69 years old) had a prostatic volume of 43.7∼79.8 mL, average 57.4 mL. Patients in both groups had obvious urination symptoms preoperatively, and urodynamic examination confirmed bladder outlet obstruction. Inclusion criteria were as follows: (1) patients aged >60 years, with progressive dyspepsia, no symptom remission after six months of proper medication, and more than once acute urinary retention; (2) the function evaluation of heart, lung, brain, and other vital organs can tolerate surgery; (3) B-ultrasound and CT diagnosis meet the BPH standard; prostate-specific antigen (TPSA) <4 ng/L. Exclusion criteria were as follows: (1) patients with severe heart and lung dysfunction; (2) severe urethral stricture; (3) diabetic patients with severe complications; (4) patients with prostate cancer; and (5) patients with long-term use of anticoagulants or hemolytic agents. In two groups, conventional resection of prostate tissue reached the prostate capsule. The removed prostate tissue was aspirated with an Ellik irrigator, and the wound was observed to have no bleeding. After the electroreception, the F20 balloon catheter was indwelled, and another F14 double cavity balloon catheter was indwelled at the cystostomy fistula in the fistula group. 500 mL of compound sodium chloride was given intravenously during the operation. If the operation time is longer than 60 min, furosemide 10–20 mg and hydroxyethyl starch 500 mL were given as appropriate. Antibiotics were routinely used to prevent infection during and after the operation. Electrosectioned prostatic debris was collected, weighed, and sent to pathological examination. The bladder was continued to be irrigated with normal saline, and blood routine and electrolytes were examined immediately before postoperative fluid replacement.

RETRACTED

### 2.2. Surgical Methods

Cystostomy: after the bladder perfusion pressure setting was completed, partial enucleation of the plasma prostate was performed in the group of these patients. The specific operation was as follows: slowly put into the electron microscope to detect whether there were abnormalities in the bladder [11]. Then from both sides of the tip of the prostate, the electric mirror shell is clockwise and counterclockwise, peel the right-left lobe of the prostate, and completely remove the prostate tissue in the left and right lower areas. Repair the wound and enucleation to stop the bleeding. Both groups of patients retained the F20 three-lumen catheter in the urethra at the end of the operation and the F16 balloon catheter at the pubic ostomy and continued bladder flushing. After surgery, the liquid from the rinse fluid recovery bucket was stirred and extracted by about 50 mL to the laboratory to determine the RBC count in the rinse fluid [12].

Robot group: (1) lymph node cleaning and control of dorsal deep vein complex; (2) open bladder neck, free vesicle: confirm the bladder neck position, open the urinary catheter to the abdominal wall, cut off the posterior bladder neck lip, find bilateral sperm tubes and break behind the prostate, and blunt combine bilateral vesicles; (3) treatment of the anterior rectal clearance, Di fascia, prostate foot, and vascular nerve bundle; (4) cut off the urethra and separate the specimen; (5) restore the continuity of the urinary tract.

### 2.3. Quality of Life Evaluation

Quality of life (QOL) was evaluated by BPHQLS, International Prostate Symptom Scale and International Prostate Quality of Life Scale (IPQOL). The total score of IPSS was 35 points, which were divided into mild symptoms (0–7 points), moderate symptoms (8–19 points), and severe symptoms (20–35 points) according to the severity.

RETRACTED

### 2.4. To Observe

Intraoperative fluid replacement volume, decreased serum sodium concentration, decreased ratio of hemocyte (HCT), decreased concentration of hemoglobin (HGB), operative time, weight of prostate resection, blood transfusion rate, postoperative fever rate (body temperature occurring once or more than once from postoperative to discharge is greater than 37.4°C), postoperative catheter blockage rate, bladder flushing time, indwelling time of catheter, and postoperative hospital stay were observed.

### 2.5. Statistical Treatment

SPSS17.0 software package was used to process the data. Measurement data were expressed as mean ± standard deviation (±*s*), and the data met the normal distribution and homogeneity of variance. An independent sample *t*-test was used to compare the surgical conditions. The scores of each scale were tested by paired sample *t*-test. The incidence of complications was compared by continuous correction *X*^2^ test, with the test level *a* = 0.05 [13].

## 3. The Results

The procedure was successfully completed in this group, and nothing was changed for any reason. PSA > 0.2 ng/ml was four weeks after 8 cases, indicating postoperative tumor residue, advanced androgen removal treatment, and further external radiotherapy at an alternative period. The other 34 cases were followed up for an average of 15.5 (10 ∼ 37) months. In the other 42 cases, the peritoneum was damaged in 4 cases during the establishment of extraperitoneal space. The average installation time of the robot was 48.5 (40 ∼ 60) min, the average operation time was 180 (150 ∼ 230) min, the average intraoperative blood loss was 298 (80 ∼ 800) ml, and 2 cases were given intraoperative blood transfusion. Total postoperative recovery feeding time was 1.7 (1∼3) d, lien catheter time was 10.7 (7∼14) d, and average hospitalization time was 10.7 (7∼14) d. Postoperative pathology reported 42 cases with prostate hyperplasia. Gleason scored ≤6: 6, 7: 5, and 9 with ≥8 points. No positive lymph nodes were found on six right sides and two bilateral.

### 3.1. Comparison of Surgical Conditions between the Two Groups

The operation time of the machine group was longer, and the difference was statistically significant. There was no statistical difference in the weight of prostatectomy between the two groups. This suggests that the surgical efficiency of the robotic group does not show an obvious advantage, but its efficiency is lower than that of the fistula group.

The cystostomy fistula was pulled out within 24 h after surgery in the experimental group, and the urethral catheters in both groups were removed 3–5 d after surgery, and the urination was clear. The patients were discharged 5–7 d after surgery. Pathological findings were consistent with nodular prostatic hyperplasia. After three months of postoperative follow-up, the operative time of the experimental group was shorter than that of the control group, and the amount of intraoperative blood loss was lower than that of the control group. The difference was statistically significant (*P* < 0.05). There were no statistically significant differences in the weight of prostate resection and the time of postoperative indwelling urethral catheterization between the two groups (*P* > 0.05) [14], as shown in Table 1.

RETRACTED

### 3.2. Comparison of RUV and Qmax before and after Operation between the Two Groups

The RUV value of the experimental group and the control group was significantly lower than that before surgery, while the Qmax value was substantially higher than that before surgery, with statistical significance (*P* < 0.05). There was no significant difference in RUV and Qmax between the two groups before and after the operation (*P* > 0.05), as shown in Table 2.

### 3.3. The Incidence of Complications in the Two Groups

No intraoperative complications such as TURS, bladder perforation, and postoperative bleeding occurred in patients of the two groups. The patients' vital signs were stable during the operation, and no abnormal heart or lung happened in the two groups. There were 2 cases of urethral stricture in both the experimental group and control group, which were cured after 3∼4 times of urethral dilation. Within one week after the operation, 3 cases in the experimental group and 2 cases in the control group developed mild urinary incontinence, which improved after strengthening anal lifting exercise. Within two weeks after surgery, one patient in the test group and six patients in the control group developed urinary tract infections, which were cured after 1OD of antibiotics according to urine bacterial culture and drug sensitivity. No complications such as bladder neck contracture, permanent urinary incontinence, and rebleeding occurred in both groups during the follow-up three months after surgery [15]. The incidence of urinary tract infection in the test group was lower than that in the control group, and the difference was statistically significant (*P* < 0.05). There was no statistically significant difference in the incidence of urethral stricture and urinary incontinence between the two groups after surgery (*P* > 0.05), as shown in Table 3.

### 3.4. Comparison of IPSS and IPQOL Scores before and after Surgery between the Two Groups

The intragroup comparison showed that the postoperative IPSS and IPQOL in the two groups were significantly lower than those before the operation, with statistical significance (*P* < 0.05). Postoperative IPSS in the experimental group was lower than that in the control group, while there was no statistically significant difference in IPQOL between the experimental group and the control group (*P* > 0.05), as shown in Table 4.

RETRACTED

### 3.5. Influence of Treatment on Each Dimension of BPHQLS

There was no difference in preoperative BPHQLS scores between the two groups. Postoperative BPHQLS scores were increased in both groups, and the difference was statistically significant (*P* < 0.05). Comparison of various dimensions showed that the improvement of disease dimension and satisfaction degree was the most obvious in the two groups, followed by physiological, social, and psychological dimensions. However, there was no statistical significance between the experimental group and the control group in each dimension after surgery (*P* > 0.05), as shown in Table 5.

### 3.6. Section

For patients with benign prostatic hyperplasia combined with bladder calculi, lithotripsy is a better choice for the treatment of bladder calculi through cystostomy access, which is not affected by the size of the patient's prostate. In addition, during the operation, the field of vision is better, and the lithotripsy efficiency is very high. The patient has more minor bladder mucosa injury, and the operation method is simple, and the operation difficulty coefficient is small. It avoids prostate bleeding caused by lithotripsy after electroreception, reduces the complications of urethral injury, hemorrhage, and urethral stricture, and dramatically reduces the operation risk. Therefore, lithotripsy with cystostomy fistula and PKRP is a scientific and safe treatment for patients with benign prostatic hyperplasia and bladder calculi.

## 4. Discussion

During TURPK, a series of pathophysiological changes and clinical manifestations, such as a large amount of hypotonic rinsing solution entering the blood circulation, cause circulation pressure to increase, cause hemodilution, and significantly decrease serum sodium, etc. When the serum sodium is lower than normal, patients may experience dizziness, nausea, irritability, and even heart failure and arrhythmia in severe cases, threatening their lives [16]. TURS is the most difficult problem for clinicians to adopt TURP. Relevant studies have shown that intraoperative suprapubic bladder puncture can reduce the occurrence of TURS by reducing intraoperative bladder pressure. The occurrence of TURS is caused by a large amount of flushing fluid entering the open vein quickly during the operation. The bladder puncture and low-pressure flushing can continue to drain so that the bladder is always in a low-pressure state, thus reducing the flow of flushing fluid into the blood and reducing the risk of surgery. In the experimental group, PKRP was performed by cystostomy, and no TURs occurred after the operation. At the same time, the method of ascending bladder microscopy through the pubic bone can ensure a clear-cutting field of vision, and the bleeding point can be found timely and accurately when there is a large amount of bleeding, it is convenient for immediate electrocoagulation to stop bleeding, and the operation time is short. The results showed that the operative time, the amount of intraoperative blood loss, and the weight of prostate resection in the experimental group were lower than those in the control group. PKRP could form a coagulation layer of 1∼3 mm on the incision surface, and the ion beam could cut the tissue faster and have a good hemostasis effect. The pathophysiological change of BPH is lower urinary tract obstruction. The urine flow rate test can be used to determine the extent of the patient's dysuria. Urine flow resistance increases, thus affecting the flow of urine. The residual urine in the bladder after urination is called residual urine volume. The pathophysiological changes of BPH are bladder outlet obstruction caused by prostatic hyperplasia and secondary detrusor function impairment. In patients with BPH, limited bladder emptied and increased surplus urine were the results of the above two factors alone or together. According to the experimental group and the control group, compared with before operation, RUV value was significantly reduced and Qmax value was significantly improved after operation, the difference was statistically significant (*P* < 0.05), bladder colostomy usually adopts four zone segmentation method, and transurethral bipolar plasma chisel method is used to partially remove the prostate, which has a significant improvement effect on patients with dysuria under normal pressure detrusor function recovery is better. The prognosis is better [9]. Due to the separation along with the prostate surgical capsule, the glandular tissue of the part of prostate hyperplasia was completely removed as far as possible, reducing the chance of BPH recurrence and also playing a certain role in improving the detection rate of accidental prostate cancer, which has a good clinical application prospect. Professor Wu Yue also reformed the PKEP operation method, which is called the cystostomy transurethral quadripartite division method for the treatment of benign prostatic hyperplasia. In other words, the prostate was artificially divided into four regions (upper region, lower right region, lower left region, and middle region), and the removal of the three regions (gouging to the area first, and then cutting the bottom right area and lower area) was performed, through the only critical areas of resection of the prostate gland, to shorten the operation time, reduce intraoperative blood loss, such as resection of the prostate weight, reduce factors of complications in patients with surgery, and improve the operation effect of urinary tract symptoms [3]. It was found that, in some surgical procedures, continuous bladder perfusion caused high pressure in the bladder, and the patient's bladder compression on the abdomen and chest affected the circulatory system and respiratory system, so it was difficult to tolerate surgery and even easy to induce cardiopulmonary adverse events, water poisoning, and other surgical complications. At the same time, due to the high bladder pressure, the rinsing fluid cannot be continuously perfused, the water flow stops, and the surgical field is not clear. The operator needs to repeatedly pull and push the electrosurgical scope to remove the excessive rinsing fluid in the bladder, which affects the operation and sometimes even forces the operation to be terminated. IPSS questionnaire is an internationally used timing scoring system for the incidence of prostate symptoms and the degree of tolerance to current symptoms. Postoperative IPSS of the experimental group was lower than that of the control group, and the difference was statistically significant (*P* < 0.05), suggesting that the severity of prostatic hyperplasia symptoms was alleviated by cystostomy and transurethral four-zone division bipolar plasma partial prostatic enucleation [17]. As one of the important indicators to evaluate the therapeutic effect, quality of life (QOL) is paramount to evaluate the therapeutic effect of the treatment of chronic diseases. Quality of life assessment can timely and accurately reflect the patient's condition, psychological, social, and satisfaction status and changes but can also reflect the patient's physical and mental health. According to the study, the prostate wound has been basically epithelialized three months after resection, and the surgical trauma has been basically recovered. Therefore, this paper conducted follow-up observation three months after resection, three months after the operation, the quality of life of the patients was greatly improved, and particularly the disease dimension was recovered. At the same time, the improvement of symptoms could eliminate the patients' troubles such as frequent urination, urgent urination, and urinary incontinence. However, there was no difference in the postoperative quality of life between the two groups. The main reason may be that both the control and test groups received electrotonic resection, which had the same effect on improving patients' symptoms, obtaining greater psychological support, and scoring the higher quality of life.

RETRACTED

## 5. Conclusions

This paper presents a method of plasma bipolar electric resection for cystostomy in treating prostatic hyperplasia in the elderly. For the specific content of this method, 42 cases of BPH patients needing surgical treatment who were admitted to the urological department of a hospital from January 2019 to March 2020 were selected. According to whether cystostomy was performed in bipolar TURP, the cystostomy group and robot group were divided into two groups. The surgical safety, surgical efficiency, complications, and nursing time between the two groups were compared. Through the experimental observation of parameter 1, suprapubic percutaneous cystostomy was performed to maintain low-pressure perfusion to remove the risk factors causing TURS, which could improve the safety of the operation and effectively excise the BPH glands, especially the BPH glands. The position of cystostomy should be appropriate, not too close to the pubic bone, so as not to collide with the resection mirror. When excising the prostate tissue, it is best not to cut into short pieces so as not to block the flushing channel and affect the operation during the operation and should be cut into strips. To prove the efficacy of plasma bipolar resection for cystostomy in the treatment of elderly prostatic hyperplasia, specifically, the results are as follows: (1) the severity of prostatic hyperplasia symptoms was reduced by cystostomy with transurethral four-zone bipolar plasma partial enucleation of the prostate. (2) It can improve the symptoms of patients, provide better psychological support, and improve the quality of life. Combined with relevant literature and the results of this study, the conclusions are summarized as follows: (1) compared with conventional pressure perfusion, low-pressure bladder perfusion can make the bladder almost empty, avoid pressing the prostate vein, save the interval fluid discharge time during traditional perfusion of pressure, and make electrocoagulation more convenient. (2) Due to the characteristics of minimally invasive suprapubic percutaneous cystostomy, patients' hospital stay can be shortened, the economic burden of patients can be reduced, and the problems of complicated and expensive medical treatment for elderly BPH patients in primary hospitals can be solved. (3) Suprapubic percutaneous cystostomy was performed under the maintenance of low-pressure perfusion to remove the risk factors causing TURS, which can improve the safety of surgery and effectively remove the BPH, especially the BPH. (4) Xinjiang is inhabited by minorities, with a large area and few people, defective medical equipment, and insufficient technical strength. There are many difficulties in carrying out electroprostatectomy or open surgery. The longer the operation time, the more significant the blood loss, which poses great risks to perioperative patients. Therefore, we need to study and pay attention to finding a relatively safe, less complicated surgical method with shorter recovery time to serve most minority patients. This research adopts low-pressure perfusion of four-region segmentation method of transurethral bipolar plasma gouge partial cutting of prostate benign BPH treatment, and it is applicable for basic-level hospitals; equipment requirements are not high (plasma cutting equipment of a complete set of about 30∼400000 yuan), and surgical skills training cycle is shorter (3∼6 months), but with the method of concentrated study and individual instruction, operation steps. The unified route ensures the safety. It can reduce the inconvenience of long-distance referral for patients, which is worth promoting in primary hospitals.

RETRACTED

## Figures and Tables

**Table 1:** Comparison of surgical conditions between the two groups.

Group	The operation time	The amount of bleeding in the book	Prostatectomy weight	Postoperative indwelling catheterization time
The control group	158.47 ± 56.86	161.00 ± 41.06	51.13 ± 17.95	79.78 ± 20.24
The experimental group	83.87 ± 22.04	98.33 ± 28.29	48.90 ± 12.26	78.79 ± 24.20
*T* value	2.024	5.866	0.479	0.136
*P* value	≤0.001	≤0.001	0.634	0.899

**Table 2:** Comparison of RUV and Qmax before and after operation between the two groups (*x* ± *s*).

Project	The experimental group		The control group	
	Before the operation	After the operation	Before the operation	After the operation
RUV	50.50 ± 15.10	13.00 ± 10.70	43.00 ± 10.06	11.00 ± 7.00
Qmax	8.07 ± 2.25	15.50 ± 8.11	7.15 ± 1.80	14.44 ± 3.33

**Table 3:** Occurrence of postoperative complications in the two groups/cases (%).

Group	The total count	Urinary tract infection	Urethral stricture	Urinary incontinence
The experimental group	36	1 (2.86)	2 (5.56)	3 (8.33)
The control group	26	6 (23.08)	2 (7.69)	2 (7.69)
*P*		<0.05	>0.05	>0.05

**Table 4:** Comparison of preoperative and postoperative IPSS and ZPQOL scores between the two groups.

Group	IPSS		*T* value	*P* value	IPQOL		*T* value	*P* value
	Before the operation	After the operation	14.329	≤0.001	Before the operation	After the operation	14.416	≤0.001
The control group	26.7 ± 3.7	8.7 ± 3.4	32.527	≤0.001	4.8 ± 0.5	1.4 ± 0.8	18.351	≤0.001
The experimental group	26.8 ± 3.4	3.8 ± 1.2			4.6 ± 0.3	1.2 ± 0.7		
*T* group	0.090	6.740			1.625	0.852		
*P* group	0.929	≤0.001			0.112	0.400		

RETRACTED

**Table 5:** BPHQLS score in each dimension of the two groups.

The dimension	The control group		*T* value	*P* value	The experimental group		*T* value	*P* value
	Before the operation	After the operation			Before the operation	After the operation		
Disease	39.2 ± 6.1	62.6 ± 6.7	10.330	≤0.001	40.3 ± 7.1	60.7 ± 7.3	10.165	≤0.001
Physiological	41.2 ± 7.0	58.4 ± 6.7	7.100	≤0.001	40.2 ± 6.0	59.3 ± 8.0	9.739	≤0.001
Social	40.7 ± 9.2	59.2 ± 7.1	6.368	≤0.001	41.7 ± 8.9	58.3 ± 9.2	7.011	≤0.001
Psychological	38.9 ± 12.1	57.4 ± 11.4	4.451	≤0.001	40.0 ± 10.7	58.3 ± 12.4	6.009	≤0.001
Satisfaction	42.2 ± 9.2	60.6 ± 8.7	5.813	≤0.001	44.3 ± 6.3	61.0 ± 9.7	7.362	≤0.001

## Data Availability

The data used to support the findings of this study are available from the corresponding author upon request.
